The article "An Updated Review of Driving-Pressure Guided Ventilation Strategy and Its Clinical Application" was published in 2022. Journal: Biomed Res Int.

# An Updated Review of Driving-Pressure Guided Ventilation Strategy and Its Clinical Application

**DOI:** 10.1155/2022/6236438

**Published:** 2022-08-02

**Authors:** Guanyu Yang, Chunhui Hu, Zhentao Sun

**Affiliations:** Department of Anesthesiology, Pain and Perioperative Medicine, The First Affiliated Hospital of Zhengzhou University, Zhengzhou 450052, China

## Abstract

Traditional lung-protective ventilation strategies (LPVS) are currently used to reduce the incidence of postoperative pulmonary complications (PPCs), including low tidal volume (VT), positive end-expiratory pressure (PEEP), low inspiratory plateau pressure (Pplat), permissive hypercapnia, and recruitment maneuver (RM). However, a meta-analysis showed that high driving pressure was closely associated with the incidence of PPCs, but not with PEEP or VT, which led to the driving pressure-guided ventilation strategy. Some studies have proved that the driving pressure-guided ventilation strategy is superior to the traditional LPVS in reducing the incidence of PPCs. The purpose of this review is to present the current research progress and application of driving pressure-guided ventilation strategy.

## 1. Introduction

Currently, most patients under general anesthesia require mechanical ventilation, which on the one hand facilitates patient management and on the other hand results in ventilator-induced lung injury (VILI) [1]. The main mechanisms of VILI include barotrauma, volutrauma, atelectrauma, and biotrauma [2], which will increase the incidence of postoperative pulmonary complications (PPCs), difficulty in extubation, prolong the length of hospital stay, and increase mortality [3]. Currently, traditional lung-protective ventilation strategies (LPVS) are routinely used to reduce the incidence of PPCs, including low tidal volume (VT), positive end-expiratory pressure (PEEP), low inspiratory plateau pressure (Pplat), permissive hypercapnia, and recruitment maneuver (RM) [4].

Many studies [5–7] have shown that traditional LPVS can reduce the incidence of PPCs. However, a meta-analysis conducted by Amato [8] showed that higher driving pressure is closely related to the incidence of PPCs, not to VT and PEEP, or only to the extent that changes in VT and PEEP affect driving pressure. Thus, a driving pressure-guided ventilation strategy was developed to minimize driving pressure during mechanical ventilation to reduce the incidence of PPCs.

In this paper, the research progress of driving pressure guided ventilation strategy in recent years is reviewed, to provide a reference for clinical mechanical ventilation and future research.

## 2. Concept and Significance of Driving Pressure

Driving pressure, defined as VT over respiratory compliance, is adjusted to counter the elastic resistance of the respiratory system to expand the chest and lungs [9]. When mechanical ventilation is performed without spontaneous respiration, the simplified calculation of the driving pressure is Pplat–PEEP (Figure 1) [10], so when the VT is set, the lower the driving pressure, the greater the compliance of the entire respiratory system. “Functional lung size” [11] refers to the ventilated lung volume at a certain VT. Ventilation above this volume will result in barotrauma, while ventilation below this volume will result in atelectasis. Respiratory compliance is maximized when ventilation is performed according to “functional lung size,” which can avoid excessive alveolar expansion or insufficient ventilation. When a driving pressure-guided ventilation strategy is used, the driving pressure can be kept at a lower level to achieve higher respiratory compliance and a “functional lung size” status. At present, the driving pressure-guided ventilation strategy is usually realized through the setting of PEEP by the simplified algorithm Pplat-PEEP of driving pressure.

## 3. Relationship between Lung Stress, Lung Strain, and Driving Pressure

Lung stress refers to the reaction force produced by the lung tissue per unit area when the tension acts on the lung tissue, the magnitude is equal to the transpulmonary pressure, but the direction is opposite [12]. Lung strain refers to the ratio of the change of lung volume to the reference lung volume during respiration; at present, functional residual capacity (FRC) is often used instead of the reference lung volume [13]. Lung stress = lung strain × *K* (specific lung elastance) [12]. The driving pressure can be divided into two parts, one is transpulmonary driving pressure and the other is cross-chest wall driving pressure. In the absence of spontaneous respiration and the patient's chest wall, elastic resistance does not significantly change, the change of transpulmonary driving pressure is the change of driving pressure [14], and the change of driving pressure reflects the change of lung stress, which has a linear relationship with lung strain. Therefore, the driving pressure can reflect the change of lung stress and lung strain, which are the important factors leading to VILI.

Protti et al. [15] experimented on the effects of different lung strains and lung stress on VILI of mechanically ventilated animals. The severity of VILI was evaluated by the change of lung weight. The results showed that the lung weight of mechanically ventilated animals did not increase when lung strain was less than 1.0, the corresponding lung stress was less than 6 cmH_2_0 when the lung strain is greater than 2.1, the corresponding lung stress is greater than 13 cmH_2_0, mechanical ventilation of animal lung weight increased significantly, and 1.0 ~ 2.1 lung strain, as well as the corresponding 6 ~ 13 cmH_2_0 lung stress is unclear, is safe or harmful. The study proves that lung stress and lung strain play an important role in the occurrence of VILI when above a certain threshold will lead to the formation of pulmonary edema.

Chiumello et al. [16] conducted a retrospective study on the correlation between driving pressure and lung stress in a total of 150 ARDS patients. Lung stress, driving pressure, and lung and chest wall elasticity were recorded at PEEP of 5 cmH_2_0 and PEEP of 15 cmH_2_0 during mechanical ventilation. The results showed that driving pressure was significantly correlated with lung stress at both levels of PEEP, and high driving pressure leads to high lung stress.

The above results indicate that the driving pressure-guided ventilation strategy can reduce lung stress and lung strain by maintaining a low driving pressure during mechanical ventilation, thereby reducing the severity of VILI and achieving the purpose of reducing PPCs.

## 4. Measurement Method of Driving Pressure

### 4.1. No Spontaneous Breathing

For mechanically ventilated patients, the simplified algorithm of driving pressure is Pplat-PEEP.

### 4.2. Spontaneous Breathing

For patients with spontaneous breathing, the pressure applied by the ventilator (Pplat-PEEP) and the pressure produced by the respiratory muscles (negative change of pleural pressure) jointly complete the inspiratory process, so the calculation method of the driving pressure is Pplat − peep + △pleural pressure [17].

## 5. Main Methods to Reduce Driving Pressure

Many clinical studies have shown that the driving pressure is closely related to PPCs, and it is recommended to maintain the driving pressure below a certain level. With the increase of driving pressure, the incidence of PPCs increases. Therefore, it is necessary to maintain a low level of driving pressure during mechanical ventilation. The following describes how to reduce the driving pressure.

### 5.1. PEEP

The simplified algorithm of driving pressure is Pplat-PEEP, so the driving pressure can be reduced by PEEP adjustment.

Ferrando et al. [18] conducted a trial on the effects of two mechanical ventilation modes on driving pressure and ventilation efficiency in 36 patients undergoing abdominal surgery. Patients in both groups were initially given 6 mL/kg of VT and PEEP of 5 cmH_2_0. After 30 minutes, both groups received RM, the control group continued with a PEEP of 5 cmH_2_0, and the other group received individualized PEEP settings. The results showed that the driving pressure of patients in the control group and the individualized PEEP group was 7.4 ± 1 cmH_2_0 vs. 5.6 ± 1 cmH_2_0 (*P* < 0.001). Compared with the control group, the dynamic lung compliance of the individualized PEEP group was increased by 22%, and the driving pressure was decreased by 28%.

Pereira et al. [19] conducted a trial of individualized PEEP during mechanical ventilation to reduce postoperative atelectasis in 40 patients undergoing abdominal surgery. The control group maintained PEEP at 4 cmH_2_0 intraoperatively. Another group of patients received individualized PEEP settings, and PEEP levels were determined by electrical impedance tomography after RM. The results showed that the driving pressure of patients in the control group and the individualized PEEP group was 11.6 ± 3.8 cmH_2_0 vs. 8.0 ± 1.7 cmH_2_0 (*P* < 0.001). The driving pressure of patients in the individualized PEEP group was lower, oxygenation was improved, and the incidence of postoperative atelectasis was reduced.

Park et al. [11] conducted a trial of the effects of conventional LPVS and driving pressure-guided ventilation strategy on the incidence of PPCs. A total of 292 patients undergoing thoracic single-lung ventilation were enrolled. The conventional LPVS group received 6 mL/kg of VT, 5 cmH_2_0 of PEEP, and RM. The driving pressure-guided ventilation strategy group accepted the same VT, RM, and set the PEEP according to the lowest driving pressure. The results showed that the median driving pressure (interquartile interval) of patients in the conventional LPVS group and the driving pressure guided ventilation strategy group were 10 (9,11) cmH_2_0 vs. 9 (8,10) cmH_2_0 (*P* < 0.001), and the incidence of PPCs was 12.2% vs. 5.5% (*P* = 0.047). The driving pressure-guided ventilation strategy can reduce the incidence of PPCs while maintaining low driving pressure during operation compared with traditional LPVS.

All the above research results showed that the PEEP setting could reduce the driving pressure, which may be the direction to choose for the PEEP of mechanical ventilation in the future.

### 5.2. VT

The definition of driving pressure is VT over respiratory compliance, and theoretically, appropriate VT can reduce driving pressure. Too much VT can cause excessive expansion of the alveoli, resulting in barotrauma and a series of inflammatory factors; too small VT can easily lead to atelectasis. At present, an individualized VT setting method is needed, but there is no related study.

## 6. Application of Driving Pressure Guided Ventilation Strategy in Different Patients

### 6.1. ARDS Patients

Pereira et al. [20] conducted a study comparing the feasibility of a ventilation strategy with limited driving pressure with conventional LPVS in patients with ARDS. Patients in the limited driving pressure group had VT of 4 ~ 8 ml/kg according to their predicted body weight (PBW), aiming a driving pressure of 10 cmH_2_0, or the lowest possible. The traditional LPVS group was ventilated according to the ARDSNet protocol, and the VT was set as 6 ml/kg according to the PBW, if the Pplat was greater than 30 cmH_2_O, the VT was adjusted to 4 ml/kg. Results showed that from the first hour to the third day, the driving pressure in the limited driving pressure group was 4.6 cmH_2_O lower than that in the conventional LPVS group (*P* < 0.001), and the VT was also lower than that of the conventional LPVS group (*P* < 0.001), it suggests that for patients with ARDS, the use of limited driving pressure ventilation strategy is feasible.

Rauf et al. [21] conducted a study on the effects of driving pressure on the morbidity and mortality of children with ARDS. Children admitted to the ICU were divided into two groups according to whether the maximum dynamic driving pressure in the first 24 hours was greater than 15 cmH_2_O. Results show that during the period of ICU, driving pressure more than 15 cmH_2_O group of children and driving pressure down to 15 cmH_2_O group of children with mechanical ventilation time median (interquartile range), respectively, 8 (6 ~ 11) vs. 5 (4 ~ 6) days (*P* < 0.001), ICU length of stay median (interquartile range), respectively, 12 (8 ~ 15) days vs. 6 days (5 ~ 8) (*P* < 0.001), more ventilator-free days at day 28 median (interquartile range) of 17 (0 ~ 22) days vs. 23 (20~24) days (*P* < 0.001). These results indicate that driving pressure less than 15 cmH_2_O can significantly decreased morbidity in children with ARDS.

### 6.2. Non-ARDS Patients

Blank et al. [22] retrospectively analyzed the mean tidal volume and driving pressure of 1019 patients with thoracic surgery during two lung ventilation and one lung ventilation. The results showed that driving pressure was a risk factor for overall postoperative morbidity (OR, 1.034; 97.5% CI, 1.001 to 1.068). The risk of major morbidity increases by 3.4% for every 1 cmH_2_O increase in driving pressure.

Neto et al. [23] meta analyzed the data of 17 RCTs, including 2250 patients, to investigate the effects of tidal volume, PEEP, and driving pressure on PPCs during mechanical ventilation. Park et al. [11] compared the effect of driving pressure-guided ventilation strategy with traditional LPVS on the incidence of PPCs in high-risk populations. Mathis et al. [24] retrospectively analyzed 4694 patients undergoing nonemergency cardiac surgery under cardiopulmonary bypass. The results of these three studies show that driving pressure was related to the development of PPCs. As the only significant mediator of LPVS, reducing driving pressure can reduce the incidence of PPCs such as pneumonia and ARDS.

These results suggest that the current driving pressure-guided ventilation strategy is more beneficial than the traditional LPVS during mechanical ventilation in both ARDS patients and non-ARDS patients. Driving pressure-guided ventilation strategy can minimize driving pressure through individualized PEEP setting, improve intraoperative oxygenation, reduce the occurrence of atelectasis and VILI, and thus reduce the incidence of PPCs.

## 7. Method of Setting the Driving Pressure Guided Ventilation Strategy

Park et al. [11] chose to set the lowest driving pressure before the incision following one-lung ventilation. The PEEP was increased from 1 cmH_2_O to 10 cmH_2_O. Each PEEP level was maintained for 10 respiratory cycles, and the driving pressure in the last respiratory cycle was recorded. The PEEP with the lowest driving pressure was eventually selected and maintained throughout the one-lung ventilation.

Spadaro et al. [25] conducted a study to compare the difference between the PEEP increasing method and the PEEP decreasing method in setting the minimum driving pressure. The PEEP increased from 0 cmH_2_O to 16 cmH_2_O in the increasing group, and the PEEP decreased from 16 cmH_2_O to 0 cmH_2_O in the decreasing group. The results show that the median driving pressure (quad interval) of the increasing and decreasing groups was 10 (9 ~ 11) cmH_2_O vs. 8 (7 ~ 11) cmH_2_O (*P* = 0.03). Patients in the decreasing group had better intraoperative oxygenation and lower driving pressure.

There is no unified driving pressure guided ventilation strategy setting method, but no matter what methods are based on the minimum driving pressure or will be driving pressure control under a certain level, at present, only a randomized controlled study shows likely to PEEP decreasing method can obtain a lower driving pressure and still need more research to confirm.

We (The First Affiliated Hospital of Zhengzhou University) currently use the PARK methods, namely, increasing PEEP to set the minimum driving pressure. But we found a defect in the process. The method is to select the driving pressure of the tenth respiratory cycle, but the driving pressure of the tenth cycle may change and be unstable because of various factors, so we made some changes. We will also increase the PEEP, but each PEEP will maintain 13 respiratory cycles, discard the first 3 respiratory cycles, start with the fourth respiratory cycle, record the corresponding Pplat of each respiratory cycle, calculate and records the corresponding driving pressure according to the simplified algorithm Pplat minus PEEP, take the highest frequency driving pressure in 10 respiratory cycles as the driving pressure corresponding to this PEEP level, and finally compare the driving pressure corresponding to 9 PEEP levels, take the minimum driving pressure corresponding to the PEEP level, and maintain this level throughout the operation.

## 8. Safe Range of Driving Pressure

In the study of Amato et al. [8], it was found that the driving pressure was less than 15 cmH_2_0 through the regulation of respiratory parameters during mechanical ventilation, and mortality of ARDS patients significantly decreased. Results of a study on outcomes in patients with ARDS conducted by Bellani [26] showed that patients with a driving pressure of more than 14 cmH_2_O on the first day of mechanical ventilation had worse outcomes.

At present, the safety range of driving pressure has not been determined, but less than 15 cmH_2_0 may be a better choice, which still needs further study to confirm.

## 9. Conclusion

Driving pressure-guided ventilation strategy is an emerging LPVS in recent years, which can be used to set individualized PEEP. Although there are still many incomplete aspects at present, its reduction in the incidence of PPCs has been confirmed by many randomized controlled studies, but more studies are needed to promote its clinical application.

## Figures and Tables

**Figure 1:** Pressure time curve of mechanical ventilation. △*P* = driving pressure = Pplat − PEEP.

## Data Availability

No new data were created or analyzed in this study. Data sharing does not apply to this article.
